# Concomitant use of renin-angiotensin system inhibitors augments the efficacy of immune checkpoint inhibitors: a systematic review and meta-analysis

This article has been retracted.

**DOI:** 10.3389/fphar.2024.1378577

**Published:** 2024-06-04

**Authors:** Junjie Yu, Fangang Meng, Wenxia Sui, Junmin Yu, Jinhai Shen

**Affiliations:** ^1^ Department of Pharmacy, The Affiliated Hospital of Qingdao University, Qingdao, Shandong, China; ^2^ Department of Pain Treatment, The Affiliated Hospital of Qingdao University, Qingdao, Shandong, China; ^3^ Center for New Drug Safety Evaluation and Research, China Pharmaceutical University, Nanjing, Jiangsu, China

**Keywords:** immune checkpoint inhibitors, renin-angiotensin system inhibitors, cancer, hypertension, meta-analysis

## Abstract

**Background:**

The impact of renin-angiotensin system inhibitors (RASIs) on the outcome of hypertensive cancer patients undergoing immune checkpoint inhibitor (ICIs) therapy remains ambiguous. This investigation sought to elucidate the consequences of RASIs use on the prognosis for this specific patient group within the context of ICIs treatment, aspiring to provide a clearer basis for rational, evidence-driven choices in the clinical prescription of these medications.

**Methods:**

A comprehensive search was conducted on PubMed, Embase, Web of Science, and the Cochrane Library for original studies published up to 6 August 2023. Studies published in English reporting hazard ratios (HRs) with 95% confidence intervals (CIs) for overall survival (OS) and/or progression-free survival (PFS) were included. All statistical analyses were executed utilizing R software (version 4.2.2).

**Results:**

A total of 13 studies, encompassing approximately 12,595 patients, satisfied the inclusion criteria. Meta-analyses demonstrated a statistically significant association between the use of RASIs and a favorable outcome in OS (HR, 0.74; 95% CI, 0.62–0.88) and PFS (HR, 0.77; 95% CI, 0.62–0.96) among cancer patients receiving ICIs treatment.

**Conclusion:**

This investigation provides compelling evidence supporting the beneficial prognostic impact of RASIs on cancer patients receiving ICIs. RASIs present a viable option as antihypertensive agents for cancer patients with hypertension undergoing ICIs treatment. Further exploration and validation through prospective studies are necessary to establish definitive guidelines for the use of RASIs in managing hypertensive cancer patients undergoing immunotherapy with ICIs.

**Systematic Review Registration:**

https://www.crd.york.ac.uk/prospero/, identifier CRD42023454886.

## 1 Introduction

Currently, immune checkpoint inhibitors (ICIs) targeting cytotoxic T lymphocyte-associated antigen-4 (CTLA-4), programmed cell death-1/ligand-1 (PD-1/L1), and lymphocyte activation gene-3 (LAG-3) have notably transformed the landscape of cancer therapy (Motzer et al., 2018; Hellmann et al., 2019; Larkin et al., 2019; Tawbi et al., 2022). While a significant proportion of patients fail to attain the expected benefits from ICIs due to various inherent and external factors (Galon and Bruni, 2019; Morad et al., 2021), there remains an unmet clinical need to identify and understand the factors that influence prognostic outcomes in ICIs therapy.

With the aging of population and advancements in anticancer therapies, hypertension has assumed a prominent position as the prevailing comorbidity among cancer patients, concurrently emerging as one of the most frequently encountered adverse events during cancer treatment (Lin et al., 2021; Cohen et al., 2023; Wang et al., 2023). In light of the intricate connection between cancer and hypertension, specialists have introduced the concept of “onco-hypertension,” underscoring the profound interweaving of physiological disturbances inherent to both diseases (Kidoguchi et al., 2021). On the one hand, inadequate control of hypertension in the oncological setting poses a dual threat, not only exacerbating the risk of cardiovascular disease and related complications, but also amplifying the susceptibility to adverse events induced by anticancer agents (Sahni, 2023). On the other hand, poorly managed hypertension can disrupt the anticancer drug regimen, leading to treatment delays or even necessitating the cessation of anticancer therapy (Tini et al., 2019). However, comprehensive clinical guidelines for managing onco-hypertension are currently absent (Cohen et al., 2023). Consequently, there exists a scarcity of evidence guiding the recommendation of appropriate antihypertensive drugs tailored for treating onco-hypertension.

Renin-angiotensin system inhibitors (RASIs), primarily comprising angiotensin-converting enzyme inhibitors (ACEIs) and angiotensin receptor blockers (ARBs), are widely acknowledged for their safety profile, therapeutic efficacy, and cost-effectiveness, making them a common choice for the management of hypertension and its associated comorbidities (Unger et al., 2020). Recently, RASIs have emerged as a pivotal modulatory agent in shaping the response to ICIs and have thus garnered considerable interest within the realm of immuno-oncology (Pinter and Jain, 2017). Preclinical investigations have demonstrated the capacity of RASIs to remodel the tumor microenvironment (TME), thereby promoting the emergence of an anticancer phenotype (Nakamura et al., 2018; Chauhan et al., 2019; Datta et al., 2023; Gu et al., 2023). In alignment with these preclinical findings, clinical studies have further corroborated the association between RASIs and immune activation (Liu et al., 2017; Boucher et al., 2023). In addition, preclinical (Datta et al., 2023) and clinical (Pinter et al., 2018) studies have consistently demonstrated that RASIs are capable of mitigating immune-related adverse events, highlighting their potential in modulating immune responses. This convergence of preclinical and clinical evidence underscores the potential therapeutic benefits of RASIs in cancer immunotherapy.

Despite numerous studies suggesting that RASIs exert immunomodulatory actions beyond their blood pressure lowering capabilities, the effect of these agents on the prognosis of hypertensive cancer patients undergoing ICIs therapy remains undetermined. Given the pressing need to identify novel strategies that can improve the efficacy of ICIs and to establish recommendations for antihypertensive drugs tailored for patients with onco-hypertension receiving ICIs, we conducted a meta-analysis to comprehensively assess the prognostic impact of RASIs in this patient population. The objective of this analysis was to provide a robust, evidence-based reference for the selection of appropriate antihypertensive drugs for this unique patient population, thereby contributing to optimized clinical outcomes.

## 2 Materials and methods

### 2.1 Protocol and guideline

This pooled analysis was conducted following the Preferred Reporting Items for Systematic Reviews and Meta-Analyses (PRISMA) guideline (Moher et al., 2009). The official protocol was registered in the systematic review registry at https://www.crd.york.ac.uk/prospero/ under the identifier PROSPERO CRD42023454886.

### 2.2 Search strategy

A comprehensive literature search was conducted by searching databases including PubMed, Embase, Web of Science, and the Cochrane Library to identify studies that could be of relevance from inception to 6 August 2023. The identification of studies involved employing Mesh terms and unstructured text in the subsequent manner: “immune checkpoint inhibitor,” “angiotensin receptor blocker,” “angiotensin-converting enzyme inhibitor,” “renin-angiotensin system,” and “cancer.” The scope of the investigation was restricted to studies published in the English, encompassing hazard ratios (HRs) accompanied by 95% confidence intervals (CIs) pertaining to overall survival (OS) and/or progression-free survival (PFS). The comprehensive search strategy is presented in Supplementary Table S1.

### 2.3 Selection criteria

Inclusion criteria were as follows: (a) patients diagnosed with solid tumors receiving ICIs; (b) reporting primary endpoints, including OS and/or PFS; (c) furnished adequate data for the computation of HR along with corresponding 95% CIs. The exclusion criteria were delineated as follows: (a) insufficient or unrelated data availability; (b) publication as either a case report or preclinical study.

### 2.4 Study selection, data extraction and quality assessment

The studies were selected and analyzed by two investigators (FM and WS). Discrepancies were deliberated with another reviewer (JY) to come to an agreement. In cases where data for both univariate and multivariate analysis model was available, the preference lay with the multivariate analysis model data. The subsequent components were obtained from each encompassed study: first author, date and category of publication, study design, number and proportion of patients subjected to RASIs, cohort size, cancer type and stage, types of RASIs, immunotherapy regimen, analytical approach, as well as HRs accompanied by 95% CIs for OS and PFS. Three separate authors (JY, FM, and WS) evaluated the quality of the included studies utilizing the modified Newcastle-Ottawa Scale (NOS) (Stang, 2010). Studies achieving NOS scores between seven and nine were categorized as high-quality research, those with scores of five or six were considered as moderate-quality, and studies achieving scores of four or less were classified as low-quality research.

### 2.5 Statistical analysis

HRs along with 95%CIs for OS or PFS were synthesized to produce a combined outcome. The heterogeneity of the included studies was assessed through the Cochrane *Q* test and *I* ^*2*^ statistic. If the *I* ^*2*^ statistic exceeds 50% and the *p*-value is less than 0.1 for the *Q* test, it was identified as substantial heterogeneity. In such cases, the random-effects model was employed for analysis. Alternatively, the fixed-effects model was utilized. A funnel plot along with Egger’s regression test was conducted to evaluate the publication bias. Sensitivity analysis was employed to assess the robustness of the results. All statistical analyses were conducted utilizing R software (version 4.2.2). Any statistical tests with a two-tailed *p*-value less than 0.05 were considered to be statistically significant.

## 3 Results

### 3.1 Study selection

Initially, a thorough search was conducted through electronic repositories, resulting in the identification of 479 potential studies. Subsequently, a rigorous selection process was undertaken to eliminate redundant entries, meticulously scrutinize the titles, and conduct a comprehensive assessment of the remaining studies (Figure 1). Finally, a total of 13 studies (Failing et al., 2016; Cortellini et al., 2020a; Cortellini et al., 2020b; Buti et al., 2021; Jain et al., 2021; Kichenadasse et al., 2021; Kostine et al., 2021; Miura et al., 2021; Pereira et al., 2021; Tozuka et al., 2021; Drobni et al., 2022; Nuzzo et al., 2022; Chiang et al., 2023) that investigated the prognostic impact of concurrent RASIs on the survival outcomes of patients undergoing ICIs were incorporated into the scope of this meta-analysis. Among the included studies, eleven were peer-reviewed articles (Failing et al., 2016; Cortellini et al., 2020a; Buti et al., 2021; Jain et al., 2021; Kichenadasse et al., 2021; Kostine et al., 2021; Miura et al., 2021; Tozuka et al., 2021; Drobni et al., 2022; Nuzzo et al., 2022; Chiang et al., 2023), while two were abstracts presented at conferences (Cortellini et al., 2020b; Pereira et al., 2021).

**FIGURE 1:** PRISMA flow diagram of study selection. HR, hazard ratio; ARBs, angiotensin receptor blockers.

### 3.2 Characteristics and quality assessment

The analysis incorporated a total of 13 studies, comprising both retrospective investigations and *post hoc* integrated analyses. These cohorts collectively involved 12,595 individuals, with OS as the primary endpoint for all, and PFS for a subset of 4,949 individuals. The demographic data revealed that approximately 5,050 patients were receiving RASIs, while roughly 7,545 patients were not. Seven of the studies focused on a diverse range of cancer types (Cortellini et al., 2020a; Cortellini et al., 2020b; Buti et al., 2021; Kichenadasse et al., 2021; Kostine et al., 2021; Drobni et al., 2022; Chiang et al., 2023). In terms of ICIs regimen, the studies encompassed a spectrum of treatment modalities, including the use of monoclonal antibodies (mAbs) targeting PD-L1/L1 or CTLA-4 alone, and combinations of mAbs targeting PD-1/L1 and CTLA-4. The NOS scores for the included studies ranged from 6 to 8, affirming a high level of methodological rigor and reliability across the board. A detailed account of the quality assessment is provided in Supplementary Table S2. The specifics regarding the attributes and outcomes of the included studies are outlined in Table 1.

**TABLE 1:** Characteristics and quality assessment results of included studies.

Studies and Pub Date	Publication type	Type of study	Country or region	No. of RASIs use/sample size (%)	Cancer type	Stage	ICIs used	RASIs used	Blood pressure in RASIs-free cohort	Analysis model	HR for OS (95% CI)	HR for PFS (95% CI)	NOS
Jain et al. (2021)	Article	RS	United States	33/178 (18.5)	UC	Metastatic	Anti-PD-(L)1	ACEIs or ARBs	NR	MVA	0.52 (0.29–0.93)	NR	7
				22/101 (21.8)	UC	Metastatic	Anti-PD-(L)1	ACEIs or ARBs	NR	MVA	0.57 (0.17–1.96)	NR	
Kostine et al. (2021)	Article	RS	France	203/635 (32.0)	Multiple	Advanced	Anti-PD-(L)1 Anti-CTLA-4	ACEIs or ARBs	NR	UVA	0.98 (0.79–1.21)	1.01 (0.83–1.23)	7
Pereira et al. (2021)	Abstract	RS	Portugal	35/127 (27.6)	NSCLC	NR	Anti-PD-(L)1 Anti-CTLA-4	ARBs	NR	NR	0.44 (0.19–1.02)	0.40 (0.17–0.93)	6
								ACEIs	NR	NR	0.75 (0.39–1.42)	0.87 (0.46–1.65)	
Buti et al. (2021)	Article	RS	Italy	66/217 (30.6)	Multiple	Advanced Metastatic	Anti-PD-(L)1 Anti-CTLA-4	ACEIs	NR	UVA	0.69 (0.48–1.01)	NR	7
Kichenadasse et al. (2021)	Article	*post hoc* analysis	Multiple	604/2539 (23.8)	Multiple	Advanced Metastatic	Atezolizumab	ACEIs, ARBs, or both	599 hypertensive patients, with 490 using other antihypertensives (including β-blockers, CCBs, diuretics)	MVA	0.92 (0.79–1.07)	0.95 (0.84–1.08)	8
Failing et al. (2016)	Article	RS	United States	11/80 (13.8)	Melanoma	Advanced	Ipilimumab	ACEIs or ARBs	21 patients on β-blockers, 13 on CCBs for hypertension	MVA	0.41 (0.10–1.71)	0.67 (0.33–1.36)	8
Miura et al. (2021)	Article	RS	Japan	40/300 (13.3)	NSCLC	Advanced	Nivolumab Pembrolizumab	ARBs	NR	UVA	0.69 (0.31–1.50)	NR	6
Nuzzo et al. (2022)	Article	RS	United States	30/100 (30.0)	RCC	Metastatic	Anti-PD-(L)1 Anti-CTLA-4	ACEIs or ARBs	NR	MVA	0.35 (0.17–0.70)	NR	7
				59/129 (45.7)	RCC	Metastatic	Anti-PD-(L)1 Anti-CTLA-4	ACEIs or ARBs		MVA	0.60 (0.34–1.06)	NR	
Tozuka et al. (2021)	Article	RS	Japan	37/256 (14.5)	NSCLC	NR	Anti-PD-(L)1	ACEIs or ARBs	43 hypertensive patients, with 40 using CCBs	UVA	0.71 (0.45–1.11)	0.59 (0.40–0.88)	7
Cortellini et al. (2020a)	Article	RS	Italy	313/1012 (30.9)	Multiple	Advanced	Anti-PD-(L)1	ACEIs or ARBs	114 patients using β-blockers	MVA	0.91 (0.74–1.11)	0.94 (0.79–1.12)	7
Drobni et al. (2022)	Article	RS	United States	3426/5910 (57.97)	Multiple	NR	Anti-PD-(L)1 Anti-CTLA-4	ACEIs or ARBs	2484 hypertensive patients: 1829 on β-blockers, 882 on CCBs	MVA	0.90 (0.84–0.98)	NR	8
Chiang et al. (2023)	Article	RS	Taiwan	171/734 (23.3)	Multiple	IV (74%)	Anti-PD-(L)1 Anti-CTLA-4	ACEIs or ARBs	192 hypertensive patients	MVA	0.50 (0.36–0.68)	0.56 (0.44–0.72)	7
Cortellini et al. (2020b)	Abstract	RS	Italy	NR/277	Multiple	Advanced	Anti-PD-(L)1	ACEIs or ARBs	NR	NR	1.14 (0.81–1.62)	NR	7

Abbreviation: ICIs, immune checkpoint inhibitors; RASIs, renin-angiotensin system inhibitors; HR, hazard ratio; OS, overall survival; PFS, progression-free survival; RS, retrospective study; UC, urothelial carcinoma; NSCLC, non-small cell lung cancer; RCC, renal cell carcinoma; NR, not report; PD-1, programmed cell death-1; PD-L1, programed cell death 1 ligand; CTLA-4, cytotoxic T lymphocyte–associated antigen 4; ACEIs, angiotensin-converting enzyme inhibitors; ARBs, angiotensin receptor blockers; CCBs, calcium channel blockers; MVA, multivariate analysis; UVA, univariate analysis; NOS, Newcastle-Ottawa Quality Assessment Scale.

### 3.3 Prognostic significance of RASIs in the pooled OS and PFS

Jain et al. (2021) and Nuzzo et al. (2022) provided prognostic outcomes for two distinct cohorts, whereas Pereira et al. (2021) reported outcomes for cohorts stratified by the type of RASIs rather than considering the entire population. Consequently, we consolidated the results from these three studies separately. Ultimately, a total of 16 cohorts reported HR data for OS, and 8 cohorts for PFS.

Given the substantial heterogeneity observed among the included studies (*I* ^*2*^ = 57% for OS and *I* ^*2*^ = 72% for PFS), a random-effects model was employed for data synthesis, thus providing a more conservative estimate of the pooled effect. The meta-analysis revealed that the combined HR was 0.74 (95% CI, 0.62–0.88) for OS and 0.77 (95% CI, 0.62–0.96) for PFS (Figure 2). Collectively, these findings suggest a noteworthy improvement in OS and PFS among hypertensive cancer patients treated with ICIs concomitantly with RASIs.

**FIGURE 2:** Forest plot of OS and PFS comparing RASIs-used and RASIs-free patients treated with ICIs. Pooled HR for OS **(A)** and PFS **(B)**. OS, overall survival; PFS, progression-frees.

### 3.4 Subgroup analysis

To identify potential sources of heterogeneity, subgroup analyses were conducted based on several key variables, including cancer type, geographical region, and analysis model.

Patients were grouped into four subcategories based on cancer type: urothelial carcinoma (UC), non-small cell lung cancer (NSCLC), melanoma, and renal cell carcinoma (RCC). Subgroup analyses disclosed that UC (HR, 0.53; 95% CI, 0.31–0.90), NSCLC (HR, 0.70; 95% CI, 0.53–0.92), and RCC (HR, 0.55; 95% CI, 0.35–0.88) subgroups experienced significantly prolonged OS (Figure 3A). Notably, no statistically significant correlation with PFS was discerned across these analyses (Figure 3B). On the other hand, the melanoma subgroups failed to demonstrate any statistically significant variations in either OS or PFS (Figure 3).

**FIGURE 3:** Forest plots of subgroup analysis stratified by cancer type. Results for OS **(A)** and PFS **(B)**. OS, overall survival; PFS, progression-free survival; HR, hazard ratio; UC, urothelial carcinoma; NSCLC, non-small cell lung cancer; RCC, renal cell carcinoma.

The cohorts were categorized into three geographic subgroups based on their regions: United States, Europe, and Asia. Subgroup analyses revealed a significant extension in OS for the United States subgroup (HR, 0.63; 95% CI, 0.46–0.86) (Figure 4A). Nevertheless, no statistically significant difference emerged in PFS within this subgroup (Figure 4B). Remarkably, the Asian subgroup showed an even greater OS extension (HR, 0.58; 95% CI, 0.44–0.78), and a similar prolongation in PFS (HR, 0.57; 95% CI, 0.46–0.70) (Figure 4). In contrast, the Europe subgroup did not show statistically significant differences in either OS or PFS (Figure 4).

**FIGURE 4:** Forest plots of subgroup analysis stratified by geographical region. Results for OS **(A)** and PFS **(B)**. OS, overall survival; PFS, progression-free survival; HR, hazard ratio.

The cohorts were bifurcated into two subgroups based on the analytical models employed. Subgroup analysis unveiled that the multivariate analysis group demonstrated significantly extended OS (HR, 0.69; 95% CI, 0.54–0.87). Conversely, the univariate analysis subgroup did not reveal a statistically significant OS difference. Additionally, neither subgroup, analyzed using multivariate nor univariate methods, demonstrated a statistically significant variation in PFS. (Supplementary Figure S1).

### 3.5 Publication bias and sensitivity analysis

The funnel plot illustrating OS displayed asymmetry in its distribution (Supplementary Figure S2A), suggesting a possible publication bias. To further assess the publication bias, we conducted an Egger’s regression test, and the significant result (*p* = 0.0068) confirmed the presence of publication bias (Supplementary Figure S2B). In addition, sensitivity analyses were undertaken to assess the robustness of the findings. The result demonstrated that the combined HR for OS remained unchanged when each individual cohort was considered, underscoring the solid reliability of the outcomes (Supplementary Figure S3A). However, the pooled PFS was affected when the study by Chiang et al. (2023) was excluded from the analysis (Supplementary Figure S3B). This suggests that the PFS data from this particular study had a significant influence on the overall pooled estimate.

## 4 Discussion

In the contemporary medical landscape, the convergence of an aging population and the advent of innovative anti-cancer therapies has led to a rise in the prevalence of hypertension among cancer patients (Kidoguchi et al., 2021). Hypertension in cancer patients, characterized by a complex interplay between hypertension and malignancy, presents significant clinical management challenges, especially due to the lack of definitive guidelines for selecting suitable antihypertensive therapies for this patient group (Cohen et al., 2023). The intricate pathophysiology linking hypertension with cancer not only increases cardiovascular risks but also complicates cancer therapy by enhancing the risk of adverse reactions and potentially disrupting treatment schedules (Sahni, 2023). RASIs, widely used in the treatment of hypertension, have been shown to possess immunomodulatory effects beyond blood pressure control (Pinter and Jain, 2017). Therefore, investigating the prognostic impact of RASIs in cancer patients with hypertension receiving ICIs holds significant clinical importance. Nevertheless, the relationship between RASIs use and the prognostic outcomes in cancer patients undergoing ICIs therapy remains clouded by inconsistent findings in the extant literature. Consequently, a comprehensive meta-analysis, consolidating evidence from diverse studies, is crucial to attain clarity on this subject. This study comprehensively assesses the prognostic impact of RASIs in cancer patients undergoing ICIs therapy via meta-analysis. Our meta-analysis incorporates a broader spectrum of cancer types and boasts a substantial patient cohort exceeding 12,000 individuals, thereby enhancing the robustness and generalizability of the findings. This enlarged scope and sample size fortify the credibility and conviction of the conclusions drawn, offering a more dependable foundation for clinical inference and future research.

To explore the sources of heterogeneity across the studies incorporated, we conducted subgroup analyses based on several key factors: cancer type, geographical region, and the analytical model applied. Our subgroup analysis revealed differential effects of RASIs across various cancer types, geographical regions and analysis models. Specifically, patients with UC, NSCLC, and RCC experienced a survival benefit, whereas those with melanoma did not. It is plausible that tumors with a naturally heightened immune response, which are known to demonstrate greater sensitivity to ICIs, may exhibit less incremental benefit from RASIs. This could stem from a ceiling effect, where the outcomes are already optimized by the inherent immune responsiveness, limiting additional improvements from RASIs. This discrepancy also encourages a nuanced exploration of how the baseline immunological profile of tumors might influence the outcomes of cancer patients undergoing ICIs therapy concomitant with RASIs. However, it is essential to also acknowledge that these agents might exert their benefits through both immunomodulatory and TME-specific mechanisms, particularly the extent of fibrosis within the TME (Diop-Frimpong et al., 2011; Jones et al., 2021; Gu et al., 2023). In addition, there is a relatively clear association between elevated blood pressure and RCC (Colt et al., 2011), hinting that blood pressure control using RASIs could have a renal vascular specific effect.

Notably, subgroup analysis revealed that cancer type is a key driver of heterogeneity. This suggests that the diverse pathophysiological profiles among distinct cancer types exert a substantial impact on the prognostic outcomes for hypertensive cancer patients undergoing concurrent treatment with ICIs and RASIs, highlighting the critical role of cancer-specific pathophysiology in determining therapeutic responses. Furthermore, the revelation highlights the inadequacy of a “one-size-fits-all” approach in managing hypertension in the context of cancer immunotherapy. Instead, it advocates for a more nuanced understanding of how individual cancer types interact with RASIs, emphasizing the need for tailored therapeutic strategies that take into account the unique tumor biology. Future translational research efforts should delve into the underlying mechanisms driving the observed heterogeneity, exploring the molecular pathways by which RASIs modulate the immune response in different cancer settings.

Furthermore, the observed regional variation, where the concurrent use of RASIs and ICIs exhibited a more pronounced effect on survival outcomes in the United States and Asia compared to Europe, suggests that diverse factors such as genetic predispositions (Ogedegbe et al., 2015), lifestyle, or differences in treatment protocols could influence the efficacy of this therapeutic approach.

The subgroup stratification based on the analytical model revealed a statistically significant prolongation of OS in the multivariate analysis subgroup, whereas the univariate analysis subgroup did not demonstrate such a significant difference. This discrepancy suggests that the multivariate approach, which considers multiple factors simultaneously, may offer a more comprehensive and accurate assessment of survival outcomes compared to the univariate approach, which focuses on individual factors alone. It implies that the survival advantage attributed to RASIs could be more nuanced, requiring careful consideration of the complex disease milieu and concurrent therapies. Collectively, these analyses underscore the importance of utilizing sophisticated statistical methods that can adequately adjust for confounders when assessing therapeutic interventions. The discrepancy between the multivariate and univariate analyses highlights the necessity for comprehensive evaluation methodologies that reflect the real-world complexity of oncological care. Future studies should consider incorporating more refined models to better elucidate the survival benefits associated with RASIs use alongside ICIs and explore the underlying mechanisms contributing to the observed differences in OS.

Despite these promising findings, there are some limitations in our study. The retrospective nature of the included studies introduces potential biases and confounding factors, which might affect the generalizability of our results to real-world clinical settings. Furthermore, the absence of comprehensive subgroup analyses, specifically pertaining to variables such as cancer stages, the line of ICIs treatment, the timing of RASIs introduction, and the specific types of RASIs used, confines our comprehension of the complete range of patient populations who could potentially derive advantage from the concurrent administration of ICIs and RASIs. Additionally, the application of Egger’s regression test revealed a significant presence of publication bias. This bias could be attributed to the tendency to publish studies with positive or significant results, while studies with negative or non-significant findings may be overlooked or delayed for publication. Therefore, we must exercise caution in interpreting and applying the findings to avoid any misleading conclusion resulting from publication bias.

Of note, it remains unclear whether initiating short-term RASIs treatment, either by transitioning to these medications upon cancer diagnosis or commencing them following a hypertension diagnosis in these patients, confers any therapeutic advantage. Therefore, investigating the optimal dosage and duration of RASIs usage, alongside exploring the molecular pathways by which RASIs enhance the efficacy of ICIs, would provide critical insights into the mechanistic underpinnings of this synergism. Future directions should involve large-scale, prospective randomized controlled trials designed to minimize bias and explore the intricacies involved in the concurrent use of ICIs and RASIs.

## 5 Conclusion

In summary, our study contributes a significant body of evidence supporting the concurrent use of RASIs with ICIs as a potential strategy to improve the prognosis of cancer patients with hypertension. While the survival benefits are evident, especially in UC, NSCLC, and RCC, the exact mechanisms and the extent to which these benefits extend across different cancers and populations remain to be fully elucidated. As such, the concurrent administration of RASIs alongside ICIs constitutes a promising area for further exploration and clinical implementation, offering hope for personalized and evidence-based management of onco-hypertension in the era of precision medicine.

## Data Availability

The original contributions presented in the study are included in the article/Supplementary Material, further inquiries can be directed to the corresponding authors.
